The article "Significance of CYP3A4∗1G and OPRM1 A118G Polymorphisms in Postoperative Sufentanil Analgesia in Women of Different Ethnicities" was retracted in 2023. Reasons: unreliable results or conclusions; concerns about the data; concerns about the peer review; concerns about the citations.

# Significance of CYP3A4∗1G and OPRM1 A118G Polymorphisms in Postoperative Sufentanil Analgesia in Women of Different Ethnicities

**DOI:** 10.1155/2022/9833591

**Published:** 2022-06-28

**Authors:** Chunying Zhang, Qiyuan Zheng, Fengting Pan, Ting Wang, Yalin Zhao, Zhaoguang Xiao, Zehan Huang

**Affiliations:** ^1^Department of Anesthesiology, Affiliated Hospital of Youjiang Medical University for Nationalities, Baise, Guangxi 533000, China; ^2^Department of Anesthesiology, Pingguo People's Hospital, Baise, Guangxi 533000, China; ^3^Department of Anesthesiology, Graduate School of Youjiang Medical University for Nationalities, Baise, Guangxi 533000, China

## Abstract

**Objective:**

To investigate the association between CYP3A4∗1G and OPRM1A118G gene polymorphisms and postoperative analgesia with sufentanil in women of Zhuang ethnicity from western Guangxi, China.

**Methods:**

Forty-eight Chinese Zhuang women who underwent elective myomectomy under general anesthesia in our hospital from January 2019 to December 2020 were selected, and another 47 Chinese Han patients in the same period were selected as the control subjects. CYP3A4∗1G and OPRM1 A118G gene polymorphisms as well as sedation and pain scores at different time points after surgery were compared between the two groups of patients to analyze the relationship between the degree of pain and dosage of sufentanil and to analyze the effect of gene polymorphisms on the occurrence of adverse reactions.

**Results:**

The frequencies of ∗1/∗1G and ∗1G/∗1G genotypes, allele 1∗G of CYP3A4∗1G and genotypes AA, and allele A of OPRM1 A118G in Zhuang patients were lower than those in Han patients, while the frequencies of ∗1/∗1, allele ∗1 of CYP3A4∗1G and genotypes AG, genotypes GG, and allele G of OPRM1 A118G were higher in Zhuang women. There was no significant difference in the Ramsay and VAS scores between the two groups at different time points after surgery, but the sufentanil use in Zhuang patients was higher than in Han patients at different time points after surgery. In addition, sufentanil use was highest in Zhuang patients with the ∗1/∗1 genotype of the CYP3A4∗1G gene. No significant difference was found in the incidence of adverse reactions during analgesia between the two groups.

**Conclusion:**

CYP3A4∗1G could be associated with postoperative sufentanil analgesia in Zhuang patients in western Guangxi and should be considered when developing personalized analgesia regimens.

## 1. Introduction

Sufentanil, a derivative of fentanyl, is one of the commonly used opioids for postoperative analgesia in China. However, scholars have found significant individualized differences in the dosage of sufentanil for postoperative analgesia and the incidence of adverse reactions after use, which may be related to the patient's genetic background [1]. Single nucleotide polymorphisms (SNPs) refer to the differences in the nucleotide sequence of a gene among individuals [2]. Previous studies have demonstrated that SNPs could lead to individualized differences in analgesic effects by affecting the pharmacokinetics of sufentanil [3]. Cytochrome P450 (CYP) 3A4 was shown to be responsible for sufentanil N-dealkylation and generation of norfentanyl, but significant differences were observed in CYP3A4 enzyme activity in different individuals [4], which may have been related to genetic factors [5].

CYP3A4∗1G is a newly discovered allele in 2014, accounting for a prevalence of 22.1% in the Han population. Studies have shown that CYP3A4∗1G gene mutation could enhance the efficacy of intravenous fentanyl in women [6], and patients with this gene mutation required a higher sufentanil dosage for analgesia 24 hours after surgery.

Sufentanil mainly acts on human *μ* opioid receptors (MOR), and in China, the OPRM1 A118G SNP has the highest incidence in encoding MOR, which produces a nonsynonymous amino acid substitution [7]. Polymorphisms at this site can cause the loss of a glycosylated site in the extracellular N-terminal region, thus seriously affecting the function of OPRM1 protein and leading to a significant decrease in the analgesic potency of sufentanil [8].

At present, there are few reports on the SNP distribution of CYP3A4∗1G and OPRM1 A118G and the relationship between their polymorphisms and postoperative sufentanil analgesia in Zhuang women in western Guangxi, China. Therefore, this study is aimed at exploring the genetic factor associated with individual differences in the analgesic effect of sufentanil, providing a scientific theoretical basis for guiding the selection of postoperative analgesia regimens for patients of different ethnic groups and different genotypes, and ultimately improving the analgesic effect and reducing the occurrence of potentially related adverse reactions.

## 2. Materials and Methods

### 2.1. Study Subjects

A total of 48 female patients of Zhuang ethnicity who underwent elective myomectomy under general anesthesia in our hospital from January 2019 to December 2020 were selected as the study subjects, and 47 Han female patients in the same period as the controls. The general data of the patients were recorded. The inclusion criteria of the study were as follows: (1) age ≥ 18 years, Zhuang nationality; (2) underwent elective myomectomy under general anesthesia and received sufentanil for analgesia 48 hours after surgery; (3) conformed to the American Society of Anesthesiologists (ASA) physical status I or II; and (4) provided informed consent and volunteered to participate in the study.

Exclusion criteria were as follows: (1) had severe heart, liver, kidney, and other organic diseases; (2) drug contraindications or drug allergy; (3) diabetes, hypertension, history of chronic pain, or use of analgesic drugs; (4) drugs that affected the CYP3A enzyme activity were taken within 1 month before surgery; (5) patients with disturbance of consciousness or mental disorders, depression, or anxiety and could not cooperate with the treatment; and (6) cases with incomplete information. This study was approved by the medical ethics committee of the Affiliated Hospital of Youjiang Medical University for Nationalities (approval no.: YYFY-LL-2019-008; Guangxi, China).

### 2.2. Anesthesia

The patients were made to fast for 8 hours and water deprivation for 4 hours before surgery. Electrocardiogram, heart rate, blood pressure, oxygen saturation, and electrical activity in the brain were observed using a monitor after entering the operating room. The patients' upper limb venous access was used for drop infusion of sodium chloride injection, and conventional oxygen inhalation was performed via a mask at an oxygen flow rate of 3 L/min. Penehyclidine hydrochloride (0.01 mg/kg) and midazolam (0.05 mg/kg) were injected 30 min before induction of anesthesia. Their heart rate, blood pressure, and oxygen saturation were recorded again after adequate analgesia.

#### 2.2.1. Induction of General Anesthesia

Propofol (0.5 mg/kg) with the effect-site concentration of 3 *μ*g/ml was intravenously injected. After the loss of consciousness, the patients were intravenously injected with remifentanil (2 g/kg) and cisatracurium besylate (0.15 mg/kg). For muscle relaxation, an intravenous injection of succinylcholine (1.5 mg/kg) was given after the patients fell asleep. Then, the patients were given mechanical ventilation at 8-10 ml/kg through orotracheal intubation.

#### 2.2.2. Maintenance of Anesthesia

With a continuous intravenous infusion of remifentanil (0.1-0.2 *μ*g/kg/min) and propofol (6-8 mg/kg/h), the depth of anesthesia was adjusted by adjusting the infusion rate. During anesthesia, in case of systolic blood pressure ≤ 80 mmHg lasting for more than 1 min, the infusion rate could be accelerated to correct hypotension. If the condition was not relieved, 5-10 mg of ephedrine was intravenously injected. The duration of anesthesia was recorded. All anesthetic drugs were stopped postoperatively, and 0.5 mg of atropine and 1 mg of neostigmine were given to antagonize the residual effects of the muscle relaxant. The patients were extubated after regaining consciousness and were assisted to normal spontaneous breathing.

### 2.3. Postoperative Analgesia

The CADD-Legacy 6300 infusion pump was used, with the drug formula for analgesia: sufentanil 0.1 mg, droperidol 5.0 mg, and normal saline added to 100 ml. Settings of patient-controlled intravenous analgesia (PCIA) were as follows: a basic dose of sufentanil: 0.5 ml/h, an additional dose of sufentanil: 2 ml/time, locking time: 5 min, the number of effective press per hour: 7 times, and maximum dose of sufentanil per hour: 145 *μ*g.

### 2.4. Outcome Measures

At 6 hours (T1), 24 hours (T2), and 48 hours (T3) after infusion of sufentanil, the analgesic effects of sufentanil and pain degree of patients were evaluated using the Ramsay scale [9] and visual analog scale (VAS) [10], respectively. The former is a 6-point scaling detailed as follows: 1 point: anxious and agitated or restless; 2 points: oriented, cooperative, and tranquil; 3 points: response to commands only; 4 points: asleep and brisk response to a light glabellar tap; 5 points: asleep and sluggish response to a light glabellar tap; and 6 points: asleep and no response to stimuli. The latter is a 10-point scale, where 0 represents no pain and 10 represents unbearable pain.

### 2.5. Incidence of Adverse Reactions

The incidence of nausea, vomiting, pruritus, and respiratory depression during analgesia was recorded for all patients, using the following formula: incidence of adverse reactions (%) = (number of cases with adverse reactions/total cases) × 100%.

### 2.6. Polymerase Chain Reaction-Restriction Fragment Length Polymorphism (PCR-RELP)

Before surgery, 3 ml of peripheral venous blood was extracted from each patient, then placed in an EDTA anticoagulant tube, and stored in a refrigerator at 4°C. Subsequently, on completion of DNA extraction from whole blood according to the instructions of the DNA extraction kit (Tiangen, China) within 7 days, the DNA was amplified using a quantitative fluorescence PCR kit (Takara, Japan). The reaction conditions of PCR were as follows: denaturation for 5 min at 94°C; 40 cycles of denaturation for 30 s at 94°C, annealing for 60 s at 60°C, extension for 60 s at 72°C, and extension for 10 min at 72°C. The PCR products were removed and stored at 4°C for testing. The primer sequences are shown in Table 1. Afterward, the amplified products were digested using MspI endonuclease (BioLabs, Singapore) and placed in a water bath for 16 h at 37°C. After that, electrophoresis was performed with a 2% gel, and digestion results were observed using a gel imager (Bio-rad, USA).

For CYP3A4∗1G, ∗1/∗1 represented wild-type, ∗1/∗1G represented heterozygous mutation, and ∗1G/∗1G represented homozygous mutation. For OPRM1 A118G, AA represented wild-type, AG/GA represented heterozygous mutation, and GG represented homozygous mutation.

### 2.7. Statistical Analysis

All analyses were performed using the SPSS 22.0 software. The *χ*^2^ test was used to evaluate whether the genotype distribution and allele distribution conformed to Hardy-Weinberg equilibrium. Continuous variables were analyzed with the *t*-test and expressed as mean ± standard deviation (mean ± SD), while categorical variables were analyzed with *χ*^2^ test and expressed as *n* (%). *P* < 0.05 was considered statistically significant.

## 3. Results

### 3.1. General Data of Patients from the Two Ethnic Groups

The general data of the patients were recorded. No significant differences were identified in height, weight, age, anesthesia time, and operation time between the two ethnic groups (Table 2, *P* > 0.05), indicating that the two groups of patients were comparable.

### 3.2. Comparison of Genotype Frequency and Allele Frequency between the Two Groups

Here, the genotype frequency and allele frequencies of CYP3A4∗1G and OPRM1A118G in the two groups were compared. Compared with Han women, Zhuang women had higher frequencies of ∗1/∗1 genotype and allele ∗1 and lower frequencies of ∗1/∗1G and ∗1G/∗1G genotypes. The frequency of allele ∗1 of the CYP3A4∗1G gene was significantly higher than that of allele ∗1G in Zhuang women (Table 3). Additionally, compared with Han women, Zhuang women had higher frequencies of AG and GG genotypes and allele G of the OPRM1 A118G gene (Table 4). Collectively, significant differences were observed between the two groups in the genotype frequency and allele frequency of CYP3A4∗1G and OPRM1 A118G (*P* < 0.05).

### 3.3. Comparison of Ramsay and VAS Scores at Different Time Points after Surgery between the Two Groups

The Ramsay score and VAS score were used to evaluate the patients' postoperative analgesic effect and pain degree, respectively. The results showed no significant difference in Ramsay score and VAS score between the Han and Zhuang patients at different time points (Figure 1).

### 3.4. Sufentanil Use at Different Time Points after Surgery in Zhuang Patients Was Greater than in Han Patients

Further analysis on the use of sufentanil between the two groups of patients at T1, T2, and T3 time points revealed a higher sufentanil consumption in Zhuang patients at all three time points (Figure 2) suggesting that sufentanil consumption could be related to CYP3A4∗1G and OPRM1 A118G genotypes.

### 3.5. Sufentanil Use Was Different in Zhuang Patients with Different Genotypes

Further, we analyzed the relationship between sufentanil consumption and different genotypes of CYP3A4∗1G and OPRM1A118G in Zhuang patients. Our results showed that sufentanil consumption was higher in patients with ∗1/∗1 genotype of CYP3A4∗1G gene compared with ∗1/∗1G and ∗1G/∗1G genotypes at T1-T3 time points. However, sufentanil consumption in Zhuang patients with different OPRM1 A118G genotypes was not significantly different at all three time points (*P* > 0.05) (Figure 3).

### 3.6. Comparison of Incidence of Adverse Reactions during Analgesia between the Two Groups

According to the statistical analysis of the incidence of adverse reactions during analgesia in the two groups, no significant difference was identified between Zhuang and Han patients (Table 5).

## 4. Discussion

Sufentanil, a N-4 thienyl derivative of fentanyl, is a highly selective MOR *μ*-receptor agonist with a high affinity to opioid receptors. It has stronger analgesic activity than morphine and fentanyl and significantly affects postoperative analgesia in patients [11, 12]. Sufentanil is characterized by significant effects on hemodynamics, long duration of action, and low incidence of adverse reactions and is widely used in postoperative analgesia. However, in practical application, individual differences were observed in the dosage and analgesic effects of sufentanil, leading to personalized analgesic management. Studies have found [13, 14] that genetic factors were a vital cause of the observed individual differences, which were closely linked to gene polymorphisms. Therefore, it is of great clinical significance to clarify the effects of gene polymorphism on the postoperative analgesic effect of sufentanil for better individualized analgesia with sufentanil.

Sufentanil was shown to cause its effect via the following process: *in vivo* absorption, liver first-pass effect, transport, reaching the target organ, and binding to the receptor for analgesia [15], in which MOR and CYP were found to be involved as well. CYP is mainly present in the endoplasmic reticulum of liver cells and the mucous membranes of the digestive system and can be involved in the metabolism of more than half of clinical drugs [16]. CYP3A4 has been confirmed to play an important role in the metabolism of sufentanil. CYP3A4∗1G (rs 2242480) in CYP3A4 intron 10 is an allele of CYP3A4. Mutations in CYP3A4∗1G are associated with decreased mRNA levels of CYP3A4, leading to a decrease in the metabolic rate of sufentanil and a relative reduction in the dosage [17]. OPRM1 A118G (rs 1799971) SNP, the most studied SNP, refers to the mutation of adenylate to guanylate at 118 bp of exon 1 [18]. OPRM1 A118G SNP results in a decrease in the number and affects the efficacy of opioids.

In this study, we detected the SNPs of CYP3A4∗1G and OPRM1 A118G in Zhuang women in western Guangxi and analyzed the correlation between their SNPs and postoperative analgesia using sufentanil. We found significant differences in genotype frequency and allele frequency of CYP3A4∗1G and OPRM1 A118G between Zhuang women and Han women. This result is consistent with that of Liang et al. [19], who suggest the presence of SNPs in CYP3A4∗1G and OPRM1 A118G genes in Zhuang and Han women. Further, no significant differences were found in Ramsay score and VAS score at different time points after surgery between the two groups. However, at different time points after surgery, our results showed that the use of sufentanil was greater in Zhuang women than in Han women, indicating that women of different ethnic groups demonstrated different requirements for sufentanil consumption to achieve the same sedation and pain levels. Further, a significant difference in sufentanil consumption among Zhuang patients with different CYP3A4∗1G genotypes was also observed. Consistent with the results of previous studies, the difference in sufentanil consumption could probably be caused by the fact that CYP3A4∗1G mutation reduces liver microsomal metabolism of sufentanil [20], causing the concentration of sufentanil in the blood to be maintained at a certain level for effective analgesia and leading to a decrease in the need for sufentanil. Zhang et al. [21] observed that sufentanil dosage in patients with CYP3A4∗1G mutant homozygotes was also reduced during analgesia after cesarean section. In contrast, we found no difference in sufentanil use in Zhuang patients with different OPRM1 A118G genotype frequencies, indicating that OPRM1 A118G genotype frequency was not associated with sufentanil use in Zhuang patients. Adverse reactions such as nausea and vomiting are common after sufentanil use in postoperative analgesia, and their incidence was shown to be related to the anesthesia methods, surgical types, and drug doses. In this study, we observed no significant difference in the incidence of adverse reactions caused by sufentanil between Zhuang and Han women and among Zhuang or Han women with different genotypes. The underlying mechanisms remain unknown and should be investigated in future studies.

Despite the interesting observations made in this study, there were some limitations. First, as this was a single-center retrospective study, further analysis using multicenter cohorts and prospective settings could provide higher evidence level findings. We only investigated 2 ethnic groups who underwent elective myomectomy in China, and patients from more painful procedures and diverse populations should be investigated in future studies. However, to limit this limitation, we tried to match the patients' baseline characteristics as far as possible. Lastly, no significant difference in the incidence of sufentanil-related adverse reactions could have been related to the relatively small sample size of this study, and therefore, further analysis with larger sample size is required.

## 5. Conclusion

The SNP of CYP3A4∗1G in Zhuang patients in western Guangxi was associated with postoperative analgesia and a lower dosage of sufentanil compared with Han patients. Therefore, patient ethnicity and CYP3A4∗1G mutation should be considered when giving postoperative sufentanil analgesia for better analgesic effects.

## Figures and Tables

**Figure 1:** Comparison of Ramsay score and VAS score at different time points after surgery between the two groups.

**Figure 2:** Comparison of sufentanil consumption at different time points after surgery between the two groups. ^∗^*P* < 0.05 and ^∗∗^*P* < 0.01 vs. Zhuang group.

**Figure 3:** Comparison of sufentanil consumption at various time points in Zhuang patients with different genotypes. ^∗^*P* < 0.05 vs. ∗1/∗1 group and ^#^*P* < 0.05 vs. ∗1/∗1G group.

**Table 1:** Primer sequences.

Gene name	Primer sequence
CYP3A4∗1G	F 5′-CACCCTGATGTCCAGCAGAAACT-3′
	R 5′-AATAGAAAGCAGATGAACCAGAGCC-3′
OPRM1 A118G	F 5′-GGTCAACTTGTCCCACTTAGATCGC-3′
	R 5′-AATCACATACATGACCAGGAAGTTT-3′

**Table 2:** General data of patients of different ethnic groups.

Group	Case (*n*)	Age (year)	Height (cm)	Weight (kg)	Anesthesia time (min)	Operation time (min)
Zhuang	48	47.27 ± 6.63	155.35 ± 6.04	55.00 ± 6.50	103.02 ± 22.02	131.08 ± 21.97
Han	47	46.21 ± 6.03	155.09 ± 1.59	55.30 ± 7.63	100.94 ± 23.85	126.74 ± 23.98

**Table 3:** Comparison of CYP3A4∗1G genotype frequency and allele frequency between the two groups.

Variables	Case (*n*)	Genotype frequency			Allele frequency	
		∗1/∗1	∗1/∗1G	∗1G/∗1G	∗1	∗1G
Zhuang	48	36 (70.5)	10 (20.8)	2 (4.2)	82 (85.4)	14 (14.6)
Han	47	23 (48.9)	19 (40.4)	5 (10.6)	65 (69.1)	29 (30.9)
*χ* ^2^		6.933			7.178	
*P*		0.031^∗^			0.007^∗^	

Note: ^∗^*P* < 0.05.

**Table 4:** Comparison of OPRM1 A118G genotype frequency and allele frequency between the two groups.

Variables	Case (*n*)	Genotype frequency			Allele frequency	
		AA	AG	GG	G	A
Zhuang	48	9 (18.8)	24 (50.0)	15 (31.3)	54 (56.3)	42 (43.8)
Han	47	21 (44.7)	19 (40.4)	7 (14.9)	33 (35.1)	61 (64.9)
*χ* ^2^		8.281			8.554	
*P*		0.016^∗^			0.003^∗^	

Note: ^∗^*P* < 0.05.

**Table 5:** Comparison of the incidence rate of adverse reactions of between the two groups.

Grouping	Gene		
	CYP3A4∗1G	OPRM1 A118G	
Zhuang (*n* = 48)	3	9	
Han (*n* = 47)	2	10	
*χ* ^2^	0.004		
*P*	0.952		

## Data Availability

The datasets used and analyzed in this study are accessible upon request from the corresponding author.

## Abbreviations

SNPs: Single nucleotide polymorphisms
CYP: Cytochrome
MOR: Human *μ* opioid receptors
ASA: American Society of Anesthesiologists
T1-3: Indicated time for measuring outcomes
VAS: Visual analog scale
PCR-RELP: Polymerase chain reaction-restriction fragment length polymorphism
SD: Standard deviation.
